# Engineering *Bacillus licheniformis* as a thermophilic platform for the production of l-lactic acid from lignocellulose-derived sugars

This article has been retracted.

**DOI:** 10.1186/s13068-017-0920-z

**Published:** 2017-10-11

**Authors:** Chao Li, Zhongchao Gai, Kai Wang, Liping Jin

**Affiliations:** 1 Clinical and Translational Research Center, Shanghai First Maternity and Infant Hospital, Tongji University School of Medicine, Shanghai, 200092 People’s Republic of China; 2 State Key Laboratory of Microbial Metabolism, and School of Life Sciences & Biotechnology, Shanghai Jiao Tong University, Shanghai, 200240 People’s Republic of China

**Keywords:** Lignocellulosic biomass, Thermophiles, *Bacillus licheniformis*, l-Lactic acid, Metabolic engineering

## Abstract

**Background:**

*Bacillus licheniformis* MW3 as a GRAS and thermophilic strain is a promising microorganism for chemical and biofuel production. However, its capacity to co-utilize glucose and xylose, the major sugars found in lignocellulosic biomass, is severely impaired by glucose-mediated carbon catabolite repression (CCR). In this study, a “dual-channel” process was implemented to engineer strain MW3 for simultaneous utilization of glucose and xylose, using l-lactic acid as a target product.

**Results:**

A non-phosphotransferase system (PTS) glucose uptake route was activated via deletion of the glucose transporter gene *ptsG* and introduction of the galactose permease gene *galP*. After replacing the promoter of glucokinase gene *glck* with the strong promoter *P*_als_, the engineered strain recovered glucose consumption and utilized glucose and xylose simultaneously. Meanwhile, to improve the consumption rate of xylose in this strain, several measures were undertaken, such as relieving the regulation of the xylose repressor XylR, reducing the catabolite-responsive element, and optimizing the rate-limiting step. Knockout of ethanol and acetic acid pathway genes further increased lactic acid yield by 6.2%. The resultant strain, RH15, was capable of producing 121.9 g/L l-lactic acid at high yield (95.3%) after 40 h of fermentation from a mixture of glucose and xylose. When a lignocellulosic hydrolysate was used as the substrate, 99.3 g/L l-lactic acid was produced within 40 h, with a specific productivity of 2.48 g/[L h] and a yield of 94.6%.

**Conclusions:**

Our engineered strain *B. licheniformis* RH15 could thermophilically produced l-lactic acid from lignocellulosic hydrolysate with relatively high concentration and productivity at levels that were competitive with most reported cases of l-lactic acid-producers. Thus, the engineered strain might be used as a platform for the production of other chemicals. In addition to engineering the *B. licheniformis* strain, the “dual-channel” process might serve as an alternative method for engineering a variety of other strains.

**Electronic supplementary material:**

The online version of this article (doi:10.1186/s13068-017-0920-z) contains supplementary material, which is available to authorized users.

## Background

Lignocellulosic biomass—one of the most abundant and attractive second-generation resources—is regarded as an economical substrate for sustainable bioprocesses [1]. Hydrolysis of lignocellulose yields a mixture of sugars, with glucose and xylose as the two main components [2]. Although the production of several biofuels and chemicals, such as ethanol, isobutanol, *n*-butanol, butane-2,3-diol (2,3-BD), and acetone, has been achieved from lignocellulose, most bacteria and yeasts cannot efficiently utilize glucose and xylose simultaneously due to the so-called carbon catabolite repression (CCR) [3, 4]. Glucose-mediated CCR always prefer sugar in the form of glucose via repressing the consumption of other sugars such as xylose, resulting in low efficiency during mixed-sugar fermentation processes [5]. Other reasons for such inefficient processes include the lack of robust genes involved in xylose metabolism or use of the hetero-phosphoketolase pathway, which leads to the generation of equal amounts of byproducts (mainly formic acid, acetic acid, and ethanol) [6]. In an effort to improve the efficiency of this process, growing attention has been devoted to engineering new strains capable of simultaneously utilizing multiple sugars.

Thermophilic microorganisms provide added benefits for the fermentation of lignocellulose-derived sugars [7]. For example, thermophilic bacteria possess highly active cellulolytic and hemicellulolytic enzymes for efficient biomass hydrolysis [8]. Meanwhile, the high-temperature process allows higher rates of feedstock conversion, minimizes the risk of contamination, lowers costs for heating and cooling, permits easier processing of feedstock, and provides opportunities for enhanced product recovery [9]. Although several thermophiles, such as *Clostridium thermohydrosulfuricum*, *Thermoanaerobacter ethanolicus*, and *B. coagulans,* can innately co-ferment pentoses and hexoses, their poor properties for using lignocellulosic biomass and the lack of optimized genetic tools have hindered their industrial application [2, 10]. For instance, most *B. coagulans* strains used for l-lactic acid production from lignocellulose-derived sugars exhibited low output [11–14] and were difficult to manipulate genetically [15]. *B. licheniformis*, a more recently developed thermophilic host, has been successfully used for the production of butane-2,3-diol (2,3-BD) [8, 16, 17], l-lactic acid [18], and d-lactic acid [9]. Unfortunately, the strain utilized cannot effectively use glucose and xylose simultaneously. Only one study described a naturally isolated *B. licheniformis* strain, X10, that could utilize glucose and xylose simultaneously for 2,3-BD production; however, this strain lacks efficient genetic tools, thereby limiting its application in biological synthesis [19].

In this work, we evaluated the derivative strain (MW3) [20] of *B. licheniformis* ATCC 14,580 for its capacity to co-utilize glucose and xylose without CCR by producing l-lactic acid, a monomer used to form biodegradable polylactic acid (PLA), as an example. Strain MW3 is a natural producer of 2,3-BD; it can efficiently produce 2,3-BD from glucose at 50–55 °C [8]. With its high cell growth rate, the capability to utilize both hexoses and pentoses, ease of genetic manipulation, and most importantly its GRAS (generally regarded as safe) status, strain MW3 is expected to function as a potential host for biotechnological applications. In a previous study, we exploited *B. licheniformis* MW3 as a thermophilic host for efficient production of polymer-grade d-lactic acid [9]. Herein, for l-lactic acid production, the genes responsible for 2,3-BD biosynthesis, *alsS* and *alsD,* were knocked out. Then, a “dual-channel” process was utilized to engineer strain MW3. First, a non-PTS glucose uptake route was activated to co-utilize glucose and xylose in strain MW3, which was then engineered to recover glucose consumption. Second, different methods were conducted to further improve the consumption rate of xylose (Fig. 1). Byproduct-producing genes, including *adhB* and *ackA,* were also knocked out to improve the l-lactic acid yield. Finally, fed-batch fermentation using lignocellulosic hydrolysate was conducted.

**Fig. 1:** Technology roadmap for l-lactic acid production from a mixture of glucose and xylose in *B. licheniformis* MW3. *Ldh* l-lactate dehydrogenase; *AlsS* α-acetolactate synthase, *AlsD* α-acetolactate decarboxylase, *XylA* xylulose isomerase, *XylB* xylulose kinase, *PtsG* glucose transporter, *GalP* galactose permease, *XylE* D-xylose transporter, *P*_*GlcK*_ promoter of gene GlcK, *PflA* pyruvate formate-lyase, *AdhB* alcohol dehydrogenase, *AckA* acetate kinase, *PPP* pentose phosphate pathway, *PTS* phosphotransferase system, *CCR* carbon catabolite repression. Red crosses indicate that genes of the pathway were deleted. Green fonts indicate the genes that were integrated into the genome of strain MW3. Green arrows indicate the pathway for co-utilization of glucose and xylose

## Methods

### Materials and chemicals

The FastPfu DNA polymerase and pEASY-Uni seamless cloning and assembly kit were acquired from Transgen Biotech (Beijing, China). The restriction enzymes were purchased from New England BioLabs (Beijing, China). The l-lactic acid (98.0%) and d-lactic acid (99.0%) standards were obtained from Sigma-Aldrich (St. Louis, MO, USA). Oligonucleotides and gene biosynthesis were performed by Sangon Biotech Co., Ltd. (Shanghai, China). Corn stover hydrolysate was kindly provided by Changchun Dacheng Group Co. Ltd. (China); the hydrolysate contained glucose (411.0 g/L), xylose (140.8 g/L), arabinose (5.0 g/L), mannose (2.4 g/L) and galactose (1.6 g/L) and was produced by washing, pulverization, steam explosion, stewing, enzymatic (cellulase) hydrolysis, and concentration. All the other chemicals and reagents were of at least analytical grade and were available commercially.

### Bacterial strains, plasmids, and culture conditions

The bacterial strains and plasmids used in this study are listed in Table 1. *Bacillus licheniformis* MW3 was kindly supplied by Meinhardt [20]. *Escherichia coli* strains DH5α and S17-1 were used for the vector construction and as the donor strain for conjugation, respectively. The vector pKVM1 carries ampicillin and erythromycin resistance genes, and temperature-sensitive replication was used for chromosomal DNA integrants [9]. Unless otherwise specified, strains were grown at 37 °C in Luria-Bertani (LB) broth (10 g/L tryptone, 5 g/L yeast extract, and 5 g/L NaCl). Ampicillin (100 μg/mL), erythromycin (5 μg/mL), and polymyxin B (40 μg/mL) were used for selection in the *E. coli* and *Bacillus* strains. X-Gal was added at 40 μg/mL for blue–white screening.

**Table 1:** Bacterial strains and plasmids used and constructed in this study

Strain and plasmid	Relevant characteristic	Source
Strain		
*Escherichia coli* DH5α	Commercial transformation host for cloning	Novagen
*E. coli* S17-1	conjugative strain able to host λ-*pir*-dependent plasmids	In lab
*B. licheniformis* MW3	*B. licheniformis* ATCC 14580 Δ*hsdR1*Δ*hsdR2*	[20]
RH01	MW3 Δ*alsS*Δ*alsD*	This study
RH02	RH01 Δ*ldh*::*ldh*_*Bc*_	This study
RH03	RH01 Δ*ldh*::*ldh*_*Bc*_ Δ*ptsG*	This study
RH04	RH01 Δ*ldh*::*ldh*_*Bc*_ Δ*ptsG*::*galP*	This study
RH05	RH01 Δ*ldh*::*ldh*_*Bc*_ Δ*ptsG*::*galP P*_*glcK*_::*P*_*als*_^a^	This study
RH06	RH01 Δ*ldh*::*ldh*_*Bc*_ Δ*ptsG*::*galP P*_*glcK*_::*P*_*als*_ Δ*xylR*	This study
RH07	RH01 Δ*ldh*::*ldh*_*Bc*_ Δ*ptsG*::*galP P*_*glcK*_::*P*_*als*_ Δ*xylR* Δ*xylA*_*Bl*_::*xylA*_*Tc*_	This study
RH08	RH01 Δ*ldh*::*ldh*_*Bc*_ Δ*ptsG*::*galP P*_*glcK*_::*P*_*als*_ Δ*xylA*_*Bl*_::*xylA*_*Bc*_	This study
RH09	RH01 Δ*ldh*::*ldh*_*Bc*_ Δ*ptsG*::*galP P*_*glcK*_::*P*_*als*_ Δ*xylA*_*Bl*_::*xylA*_*Tx*_	This study
RH10	RH01 Δ*ldh*::*ldh*_*Bc*_ Δ*ptsG*::*galP P*_*glcK*_::*P*_*als*_ Δ*xylA*_*Bl*_::*xylA*_*Tc*_	This study
RH11	RH01 Δ*ldh*::*ldh*_*Bc*_ Δ*ptsG*::*galP P*_*glcK*_::*P*_*als*_ Δ*xylA*_*Bl*_::*xylA*_*Ml*_	This study
RH12	RH08 Δ*pflA*	This study
RH13	RH08 Δ*adhB*	This study
RH14	RH08 Δ*ackA*	This study
RH15	RH08 Δ*adhB*Δ*ackA*	This study
Plasmid		
pKVM1	Gene knockout vector, OriT, *traJ*, *ery* ^*r*^ *, amp* ^*r*^	[9]
pKVM01	For deletion of *alsS* and *alsD* genes of strain MW3	This study
pKVM02	For replacement of *ldh* gene of strain RH01 with *ldh*_*Bc*_	This study
pKVM03	For deletion of *ptsG* gene of strain RH02	This study
pKVM04	For replacement of *ptsG* gene of strain RH02 with *galP*	This study
pKVM05	For replacement of *P*_*glcK*_ of strain RH04 with *P*_*als*_	This study
pKVM06	For deletion of *xylR* gene of strain RH05	This study
pKVM07	For replacement of *xylA*_*Bl*_ gene of strain RH06 with *xylA*_*Tc*_	This study
pKVM08	For replacement of *xylA*_*Bl*_ gene of strain RH05 with *xylA*_*Bc*_	This study
pKVM09	For replacement of *xylA*_*Bl*_ gene of strain RH05 with *xylA*_*Tx*_	This study
pKVM10	For replacement of *xylA*_*Bl*_ gene of strain RH05 with *xylA*_*Tc*_	This study
pKVM11	For replacement of *xylA*_*Bl*_ gene of strain RH05 with *xylA*_*Ml*_	This study
pKVM12	For deletion of *pflA* gene of strain RH08	This study
pKVM13	For deletion of *adhB* gene of strain RH08	This study
pKVM14	For deletion of *ackA* gene of strain RH08	This study

^a^ *P*_*glcK*_ promoter of glucokinase gene *glcK*

For seed culturing, *B. licheniformis* was maintained at 4 °C on a GSY agar slant [21], which contains 10 g/L yeast extract, 5 g/L soybean peptone, 20 g/L glucose and 10 g/L CaCO_3_. The fermentation medium contained 10 g/L yeast extract, 5 g/L soybean peptone, and different concentrations of glucose and/or xylose or lignocellulosic hydrolysates. In short, for xylose fermentation, the initial concentration of xylose was approximately 57.0 g/L. For mixed-sugar fermentation, the initial concentration of glucose and xylose were approximately 60.0 and 20.0 g/L, respectively, in both batch and fed-batch fermentations. The seed culture was prepared as follows: a loop of cells from a fully grown slant was inoculated into a 100-mL Erlenmeyer flask containing 30 mL of GSY medium and was incubated statically at 50 °C for 24 h. The seed culture was then amplified in an Erlenmeyer flask with an inoculum volume of 10% (v/v).

### Genetic manipulation in *B. licheniformis* MW3

All primers used for construction are listed in supplementary Table S1, and the constructed plasmids and strains are listed in Table 1. The DNA fragment (termed as *P*_als_) upstream of the start codon (300 bp) of the *alsS* gene (GenBank: 52350029) from *B. licheniformis* MW3 was used. The genes encoding thermophilic xylose isomerase (*xylA*) were from *B. coagulans* 36D1 (termed as *xylA*_*Bc*_; GenBank: AEO99969), *Thermoanaerobacterium xylanolyticum* (termed as *xylA*_*Tx*_; GenBank: WP_013788598), *Thermobacillus composti* (termed as *xylA*_*Tc*_; GenBank: WP_015253490), and *Muricauda lutaonensis* (termed as *xylA*_*Ml*_; GenBank: WP_045800855), respectively. The *ldh*_*Bc*_ gene encoding thermophilic l-lactate dehydrogenase was from *B. coagulans* 2–6. All four *xylA* genes were codon-optimized (Text 1) for *B. licheniformis* ATCC 14580 and were synthesized by Sangon Biotech Co., Ltd.

To knock out *alsS* and *alsD* (GenBank: 52350028), the flanking regions 749 bp upstream and 659 bp downstream were amplified using the primer pairs AlsSD-up-F/AlsSD-up-R and AlsSD-dn-F/AlsSD-dn-R and were then seamlessly assembled into the *Eco*RI/*Bam*HI sites of plasmid pKVM1, resulting in plasmid pKVM01 (Figure S1A). Similarly, the vectors for deletion of genes *ptsG*, *xylR*, *pflA*, *adhB*, and *ackA* were constructed and called pKVM03, pKVM06, pKVM12, pKVM13, and pKVM14, respectively (Additional file 1: Figure S1C, F, L, M, and N).

To construct the vector for the replacement of the *ldh* gene with *ldh*_*Bc*_, the flanking regions 737 bp upstream and 667 bp downstream of the *ptsG* gene were amplified from the genomic DNA of strain MW3 using the primer pairs Ldh-up-F/Ldh-up-R and Ldh-dn-F/Ldh-dn-R. These two flanking regions were ligated along with *ldh*_*Bc*_ (cloned from *B. coagulans* 2–6 using primer pairs Ldh-F/Ldh-R) into the *Eco*RI/*Bam*HI sites of plasmid pKVM1 via the seamless cloning and assembly method, creating pKVM02 (Additional file 1: Figure S1B). Plasmids pKVM04, pKVM05, pKVM07, pKVM08, pKVM09, pKVM10, and pKVM11 were generated using the same procedure as for pKVM02 (Additional file 1: Figure S1B, D, E, G–K).

*Escherichia coli* S17-1 cells harboring pKVM plasmids were used as the donors in conjugation with *B. licheniformis* MW3. The conjugation and gene knockout with pKVM plasmids were performed as described previously [22]. All the deletion and insertion mutations were verified by PCR amplification of the genomic DNA with appropriate primers, followed by sequencing of the amplified products.

### Enzyme activity assays

To assay the enzymatic activities of the crude extracts, strains were grown for 12 h, and cells were harvested via centrifugation (8000×*g*, 10 min), washed twice with 50 mM PBS buffer (pH 7.0), and resuspended in the same buffer. The cells were then disrupted by sonication in an ice bath. The cell extract was centrifuged at 14,000×*g* for 30 min at 4 °C, and the supernatant was used for the enzyme assay. Total protein concentration was determined according to the method of Bradford using bovine serum albumin as the standard [23]. The activities of l- and d-LDH were assayed in a reaction mixture containing 50 mM pyruvate, 20 mM NADH and 0.1 mg/mL cell extracts for 10 min. Thereafter, the LDH activities were inactivated by boiling for 5 min. Then, l-lactic acid and d-lactic acid were detected by HPLC with a chiral column. The l- and d-LDH activities in *B. licheniformis* strains were calculated according to the corresponding concentrations of l- and d-lactic acid [24]. One unit of protein activity was defined as the amount of enzyme that catalyzed the consumption of 1 μmol NADH per minute, as previously described [9].

### Batch and fed-batch fermentations

The fermentations were conducted in a 5-L bioreactor (BIOSTAT B, B. Braun Biotech International GmbH, Germany) containing 2.5 L of fermentation medium. The seed culture prepared was inoculated (10%, v/v) into the fermentation medium. The cultivation was conducted at 50 °C and 80 rpm. The pH was maintained at 7.0 by the automated addition of 25% (w/v) Ca(OH)_2_. In fed-batch fermentation, a mixture of glucose and xylose (ratio of glucose to xylose approximately 3:1) or corn stover hydrolysate (700 g/L of sugars) was fed into the bioreactor to maintain the sugar concentration when the reducing sugar concentration was below 20.0 g/L. Samples were collected periodically to determine the cell density and concentrations of sugar, l-lactic acid, and byproducts.

### Analytical methods

2,3-BD was analyzed using a gas chromatograph (GC; GC2014c, Shimadzu). Samples were centrifuged at 12,000×*g* for 10 min and were then extracted with an equal volume of ethyl acetate after the addition of benzyl alcohol as the internal standard. The GC system was equipped with capillary GC columns (AT SE-54; inside diameter, 0.32 mm; length, 30 m; Chromatographic Technology Center, Lanzhou Institute of Chemical Physics, China), and nitrogen was used as the carrier gas. The injector temperature and detector temperature were both 280 °C. The column oven was maintained at 40 °C for 3 min, after which it was programmed to increase to 80 °C at a rate of 1.5 °C/min. The temperature was then raised to 86 °C at a rate of 0.5 °C/min and finally to 200 °C at a rate of 30 °C/min. The injection volume was 1 μL.

The concentrations of glucose, xylose, and fermentation products, including lactic acid, formic acid, acetic acid, succinic acid, and ethanol, were measured in an HPLC (Agilent 1200 series, Hewlett-Packard, USA) equipped with a Bio-Rad Aminex HPX-87H column (300 × 7.8 mm) and a refractive index detector. Analysis was performed with a mobile phase of 5 mM H_2_SO_4_ at a flow rate of 0.5 mL/min at 55 °C. Stereoselective assays of l-lactic acid and d-lactic acid were performed in an HPLC equipped with a chiral column (MCI GEL CRS10 W, Japan) and a tunable UV detector at 254 nm. The mobile phase was 2 mM CuSO_4_ at a flow rate of 0.7 mL/min and 25 °C. The optical purity of d-lactic acid was described as the enantiomeric excess (ee) value, defined as [(d-lactic acid) − (l-lactic acid)]/[(d-lactic acid) + (l-lactic acid)] × 100%.

## Results

### Construction of an l-lactic acid producer from *B. licheniformis* MW3 and its utilization of xylose

*B. licheniformis* MW3 is a natural producer of 2,3-BD. To produce l-lactic acid in this strain, the genes responsible for 2,3-BD synthesis (*alsS* and *alsD*) were knocked out (Table 1, Additional file 1: Figure S1). The resulting strain, designated RH01, was used to test the biosynthesis of l-lactic acid from xylose. Fed-batch fermentation was performed in a 5-L fermenter with an initial xylose concentration of approximately 55 g/L [19]. In our previous study, d-lactic acid production by strain MW3 was distinctly affected by the pH of the incubation medium and exhibited a maximum productivity at pH 7.0 [9]. Thus, in this study, pH 7.0 was chosen for the engineered strain RH01. As shown in Fig. 2a, no 2,3-BD was detected in RH01, and 73.4 g/L l-lactic acid was obtained from 113.1 g/L xylose after 62 h. The productivity was 1.2 g/[L h], and the yield was 64.9% of the theoretical yield. The concentrations of acetic acid, ethanol, and succinic acid were 6.7, 5.5, and 0.31 g/L, respectively. A large amount of formic acid (20.1 g/L) was detected in the medium, suggesting that the native l-lactate dehydrogenase (LDH) might not be sufficiently robust to compete with other enzymes in consuming pyruvate.

**Fig. 2:** Time-course of fed-batch fermentation by strains RH01 and RH02 from xylose. **a** RH01; **b** RH02. The fermentations were conducted in a 5-L bioreactor with 2.5 L of initial medium. The initial concentration of xylose was approximately 57.0 g/L. The cultivation was performed at 50 °C with stirring at 80 rpm. The pH was maintained at 7.0 by automatic addition of 25% (w/v) Ca(OH)_2_. Xylose was added to the medium when its concentration was lower than 20.0 g/L. Each fermentation condition was repeated at least twice, and typical fermentation kinetics are shown here

To verify this assumption, LDH activity in the crude extract of strain RH01 was tested. As expected, a relatively low LDH activity of 0.31 U/mg was observed. To enhance LDH activity, the native LDH encoding gene *ldh* (GenBank: AAU39324) was replaced with *ldh*_*Bc*_ (GenBank: AEH52590) from a thermophilic l-lactic acid-producer *B. coagulans* 2–6 [25] to construct strain RH02 (Table 1, Additional file 1: Figure S1). As shown in Fig. 2b, both the l-lactic acid titer (96.9 g/L) and yield (85.2%) of strain RH02 expressing *ldh*_*Bc*_ were higher than those of RH01. Increased LDH activity (0.94 U/mg) was also detected in this strain, which might have helped to divert the carbon flux of the major byproduct, formic acid, to the formation of l-lactic acid. In addition, the concentrations of acetic acid, ethanol, and succinic acid were significantly decreased (Table 2). Thus, the results suggested that strain RH02 could efficiently use xylose and might be a good candidate for the production of enantiopure l-lactic acid from lignocellulosic hydrolysates.

**Table 2:** Cell growth, sugar consumption, products, and LDHs activities of different strains

Strain	Cell density (OD_600_)	Sugar consumed (g/L)			Products (g/L)					Yield (%)	Activity of LDHs
		Glucose	Xylose	Glucose + xylose	l-Lactic acid	Formic acid	Acetic acid	Succinic acid	Ethanol		
RH01^a^	6.7	–^b^	113.1	–^b^	73.4	20.1	6.7	0.31	5.5	64.9	0.31
RH02^a^	7.2	–^b^	113.7	–^b^	96.9	6.7	4.3	0.22	3.2	85.2	0.94
RH02	7.5	58.6	0.72	59.4	53.3	1.7	2.1	< 0.1	1.5	89.7	ND^c^
RH03	6.6	33.5	13.4	46.9	41.3	1.9	1.8	< 0.1	1.4	88.1	ND^c^
RH04	6.9	51.8	12.5	64.3	56.4	2.5	2.7	< 0.1	1.8	87.7	ND^c^
RH05	7.2	57.0	12.3	69.2	61.1	2.5	2.8	< 0.1	1.8	88.3	ND^c^
RH06	7.4	57.3	14.2	71.5	63.2	2.6	2.8	< 0.1	1.9	88.4	ND^c^
RH07	7.0	56.2	13.2	69.4	60.9	2.6	2.6	< 0.1	1.8	87.8	ND^c^
RH08	7.8	57.1	18.0	75.0	66.7	2.7	2.7	< 0.1	2.1	88.9	ND^c^
RH09	7.4	56.9	15.1	72.0	64.2	2.5	2.9	< 0.1	1.8	89.2	ND^c^
RH10	7.1	56.2	13.8	70.0	62.2	2.6	2.6	< 0.1	1.9	88.9	ND^c^
RH11	6.9	56.4	13.4	69.8	61.8	2.8	2.7	< 0.1	1.8	88.5	ND^c^

The experiments were conducted in 5-L bioreactor with 2.5 L initial medium at 50 °C for 29 h. The initial concentration of mixture sugars was 80 g/L (glucose:xylose = 3:1, w/w). The cultivation was carried out at 50 °C, stirring at 80 rpm. The pH was maintained at 7.0 by automatic addition of 25% (w/v) Ca(OH)_2_ using a program-controlled peristaltic pump

^a^The experiments were carried out only using xylose for 62 h

^b^Not exist

^c^Without measurement

### Co-utilization of glucose and xylose by engineered *B. licheniformis* MW3

Hydrolysis of lignocellulose, such as corn stover, generates a solution primarily consisting of glucose and xylose at a ratio of approximately 3:1 (w/w) [1]. Thus, we tested the capability of strain RH02 to ferment a mixture of glucose and xylose (3:1, w/w). Strain RH02 used glucose preferentially over xylose, the latter of which could hardly be consumed when glucose was present (Fig. 3a, Table 2). As a result, only 0.72 g/L of xylose was consumed at the end of the fermentation. To eliminate CCR, we constructed strain RH03 by the deletion of the *ptsG* gene (GenBank: AAU40497), which encodes the major glucose transporter EIICBA in PTS in strain RH02 (Table 1, Additional file 1: Figure S1). As shown in Fig. 3b, although strain RH03 could use glucose and xylose simultaneously, the gene deletion has slowed the cell growth and l-lactic acid production upon glucose. After 29 h of fermentation, up to 13.4 g/L xylose was consumed, with 26.5 g/L glucose remaining (Table 2).

**Fig. 3:** Time course of batch fermentation by *B. licheniformis* strains RH02, RH03, RH04, and RH05 from a glucose and xylose mixture (3:1). **a** RH02; **b** RH03; **c** RH04; **d** RH05. The fermentations were conducted in a 5-L bioreactor with 2.5 L of initial medium. The initial concentrations of glucose and xylose were approximately 60.0 and 20.0 g/L, respectively. The cultivation was performed at 50 °C with stirring at 80 rpm. The pH was maintained at 7.0 by automatic addition of 25% (w/v) Ca(OH)_2_. Each fermentation condition was repeated at least twice, and typical fermentation kinetics are shown here

To recover glucose consumption, the previously reported galactose permease encoded by the *galP* gene (GenBank: AFM61492) [1] was integrated into the genome locus of *ptsG* of strain RH03 (Table 1, Additional file 1: Figure S1). The resulting strain, RH04, exhibited significantly enhanced glucose consumption and l-lactic acid production rates. As a result, 56.4 g/L l-lactic acid was produced via the consumption of 51.8 g/L glucose and 12.5 g/L xylose (Fig. 3c, Table 2). It can be seen that the consumption rate of glucose was slow compared with that of strain RH02. To further resolve this point, the promoter of the glucokinase gene *glck* (GenBank: AAU41533) was substituted with the strong promoter P_als_ from the 2,3-BD gene cluster to construct strain RH05 (Table 1, Additional file 1: Figure S1). As shown in Fig. 3d, strain RH05 used glucose more rapidly and had a consumption rate similar to that of strain RH02. The final concentration of l-lactic acid produced by RH05 was 61.1 g/L, which was 47.9% higher than that of strain RH03 (Table 2).

### Further enhancement of xylose utilization via engineering of the xylose metabolic pathway

The xylose assimilation pathway enables the isomerization of xylose to xylulose followed by phosphorylation to xylulose-5-phosphate, which is encoded by the *xyl* operon, containing xylose repressor (*xylR*, AAU42862), xylulose isomerase (*xylA*, AAU42861), and xylulose kinase (*xylB*, AAU42860). Although strain RH05 can use glucose and xylose simultaneously, the consumption rate of xylose was still relatively low, especially after recovering the glucose utilization compared with strain RH03 (Table 2). It has been reported that XylR could specifically repress the d-xylose pathway genes in some Gram-positive organisms [26]. To enhance xylose utilization in strain RH05, the gene *xylR* was deleted (Table 1, Additional file 1: Figure S1). As shown in Table 2, only a slight increase in xylose utilization was noted in the mutant strain RH06, indicating that deregulation of XylR-mediated repression could not enhance the xylose consumption rate.

Considering that the transcription of the *xyl* operon is also catabolite-repressed by the *cis*-acting catabolite-responsive element (CRE) located in the *xylA* gene in *Bacillus* sp. [27], the *xylA* gene from strain RH06 was replaced with *xylA*_*Tc*_ (GenBank: WP_015253490) from a thermophilic Gram-negative (GN) *Thermobacillus composti*. However, the utilizations of both glucose and xylose were slower in mutant strain RH07 than in strain RH06. The result suggested that optimization through substituting the GN-derived *xylA*_*Tc*_ was not effective at lifting the catabolite repression in *B. licheniformis* (Table 2).

Having determined that the xylose isomerase was the rate-limiting step in the xylose catabolic pathway and that improving the xylose isomerase-based xylose catabolic pathway can effectively strengthen both the cell growth rate and the xylose consumption rate [28, 29], we then assessed varied xylose isomerases from both Gram-positive (GP) and Gram-negative (GN) thermophilic bacteria. In brief, *xylA* in strain RH05 was replaced with *xylA*_*Bc*_ (GP; GenBank: AEO99969) of *B. coagulans*, *xylA*_*Tx*_ (GP; GenBank: WP_013788598) of *Thermoanaerobacterium xylanolyticum*, *xylA*_*Tc*_ (GN; GenBank: WP_015253490) of *T. composti*, and *xylA*_*Ml*_ (GN; GenBank: WP_045800855) of *Muricauda lutaonensis* to generate strains RH08, RH09, RH10, and RH11, respectively (Table 1, Additional file 1: Figure S1). As shown in Table 2, all four of the strains used xylose more rapidly and produced more l-lactic acid. Strain RH08 showed the highest xylose utilization, with a 46.3% increase (from 12.3 to 18.0 g/L), and produced 66.7 g/L l-lactic acid, more than was produced by the other strains. The yield of l-lactic acid and the byproducts produced by strain RH08 were comparable to or better than those obtained with strains RH09, RH10, RH11, and RH05. Thus, strain RH08 was selected for subsequent experiments.

### Byproduct elimination

For strain RH08, the major byproducts were obtained as formic acid (2.7 g/L), ethanol (2.1 g/L) and acetic acid (2.7 g/L). To enhance the L-lactic acid yield on glucose-xylose in this strain, we tried to block the biosynthetic pathways of the byproducts via gene deletion. The gene *pflA* (GenBank: AAU41018) encoding a pyruvate formate-lyase for formic acid formation was knocked out. As shown in Table 3, although less than 0.1 g/L of formic acid was detected in the resultant strain RH12, the cell growth and sugar utilization of the mutant strain were both slowed. In contrast, strain RH13, with a deletion of *adhB* (encoding alcohol dehydrogenase; GenBank: AAU42647), produced no ethanol, and strain RH14, with a knockout of *ackA* (encoding acetate kinase; GenBank: AAU41949), produced only 0.51 g/L acetic acid; meanwhile, cell growth and l-lactic acid production were negligibly affected by disruption of the ethanol and acetic acid biosynthetic pathway genes. After eliminating both *adhB* and *ackA* genes, the yield of l-lactic acid produced by the new strain RH15 increased from 88.9 to 95.1%, and only a small amount of formic acid was observed as the main byproduct, rendering strain RH15 a good candidate for l-lactic acid fermentation.

**Table 3:** Effect of different genes knocked out on l-lactic acid production

Strain	Cell density (OD_600_)	Sugar consumed (g/L)			Products (g/L)					Yield (%)
		Glucose	Xylose	Glucose + xylose	l-Lactic acid	Formic acid	Acetic acid	Succinic acid	Ethanol	
RH08	7.8	57.1	18.0	75.0	66.7	2.7	2.7	< 0.1	2.1	88.9
RH12	4.9	42.8	13.5	56.3	50.3	< 0.1	2.0	< 0.1	1.6	89.3
RH13	8.0	57.8	18.1	75.9	68.5	2.8	3.0	< 0.1	< 0.1	90.3
RH14	7.6	56.2	17.6	73.8	68.2	2.9	0.51	< 0.1	2.4	92.4
RH15	7.7	56.3	17.8	74.1	70.5	3.1	0.12	< 0.1	< 0.1	95.1

The experiments were conducted in 5-L bioreactor with 2.5 L initial medium at 50 °C for 29 h. The initial concentration of mixture sugars was 80 g/L (glucose: xylose = 3: 1, w/w). The cultivation was carried out at 50 °C, stirring at 80 rpm. The pH was maintained at 7.0 by automatic addition of 25% (w/v) Ca(OH)_2_ using a program-controlled peristaltic pump

### Fed-batch fermentation of glucose and xylose

To reduce the probable inhibitory effects of high substrate concentrations and to achieve a higher l-lactic acid concentration, fed-batch fermentation was conducted in a 5-L fermenter using strain RH15. The initial total sugar concentration used was approximately 80 g/L. As shown in Fig. 4a, 121.9 g/L of l-lactic acid (purity > 99.7%; see Additional file 1: Figure S2) was obtained from 97.4 g/L glucose and 30.5 g/L xylose after 40 h of fermentation, resulting in a l-lactic acid productivity of 3.05 g/[L h] and a yield of 95.3% of the theoretical yield. The concentration of formic acid increased to 8.2 g/L in the first 14 h and then decreased to 4.3 g/L at 40 h. The concentration of acetic acid was less than 0.2 g/L, while ethanol and succinic acid were not detected at the end of the fermentation.

**Fig. 4:** Time course of fed-batch fermentation of l-lactic acid by *B. licheniformis* strain RH15. **a** Mixed-sugar (glucose: xylose = 3:1) was used as a substrate; the initial concentrations of glucose and xylose were approximately 60.0 and 20.0 g/L, respectively; **b** Corn stover hydrolysate was used as the substrate. The fermentations were conducted in a 5-L bioreactor with 2.5 L of initial medium. The cultivation was performed at 50 °C with stirring at 80 rpm. The pH was maintained at 7.0 by automatic addition of 25% (w/v) Ca(OH)_2_. Mixed sugar (the ratio of glucose to xylose was approximately 3:1) or corn stover hydrolysate (700 g/L of sugars) was added to the medium when the glucose concentration was lower than 20.0 g/L. Each fermentation condition was repeated at least twice, and typical fermentation kinetics are shown here

### Fed-batch fermentation of corn stover hydrolysate

Corn stover hydrolysate (CSH), as one of the most popular lignocellulosic hydrolysates, was selected for l-lactic acid fermentation with an initial sugar concentration of approximately 80 g/L. CSH was supplemented to maintain the sugar concentration throughout the fermentation process once the concentration of glucose fell below 20 g/L. As shown in Fig. 4b, 99.3 g/L of l-lactic acid (purity > 99.7%) was obtained with consumption of 79.9 g/L glucose and 25.1 g/L xylose after 40 h. The productivity was 2.48 g/[L h], and the yield was 94.6% of the theoretical yield.

## Discussion

In this study, we established *B. licheniformis* MW3 as a platform for l-lactic acid production from lignocellulose-derived sugars. A “dual-channel” process was used to engineer the metabolic pathways of glucose and xylose successively. Although the constituent metabolic engineering strategies have been demonstrated for enhancing glucose and/or xylose utilization in strains such as *Corynebacterium glutamicum* [30], *Enterobacter cloacae* [1], *Saccharomyces cerevisiae* [28], and *B. subtilis* [27], they have not been used for enhancing l-lactic acid production from glucose and xylose, nor have they been studied in *B. licheniformis* previously. Using our new combinatorial “dual-channel” process, the engineered strain, RH15, was capable of producing 121.9 or 99.3 g/L l-lactic acid after 40 h fermentation from a mixture of glucose and xylose or from lignocellulosic hydrolysate, indicating that the strategy was functional and effective.

As is commonly known, CCR can severely impair the co-utilization of glucose and xylose and can result in a low mixed-sugar fermentation yield. To address the problem of inefficient utilization, various metabolic engineering strategies have been implemented in recent years. These strategies mainly include substituting PTS with inositol permeases (*iolT1*) and glucokinase (*glk*), overexpressing ATP-forming phosphoenolpyruvate carboxykinase to increase ATP supply, and incorporating heterologous xylose catabolism genes, such as the d-xylose-proton symporter (*xylT*), *xylA* and *xlyB*, and the pentose transport gene *araE* [3, 30–32]. These methods can greatly reduce the CCR and enhance the titers and yields of the products. Herein, we showed that the integration of *galP* and replacement with the strong promoter *P*_als_ could effectively enhance the glucose consumption rate by 54.6 and 10.2%, respectively, after eliminating CCR. Both results were in accordance with previous reports [1, 31], indicating that GalP and *P*_als_ were also functional in *B. licheniformis* for glucose utilization. The inactivation of *xylR* also played a weak role in promoting the xylose consumption rate, possibly because the relieved repression from XylR was unable to significantly improve the expression of d-xylose pathway genes. Furthermore, XylA derived from GP strain were more efficient in optimizing the rate-limiting step compared with those from GN strains, suggesting the different sensitivities to gene expression in GP and GN strains [33, 34].

l-Lactic acid is produced from pyruvic acid in a mixed-acid fermentation process involving several byproducts, such as formic acid, acetic acid, ethanol, and succinic acid [9]. The increased byproducts not only lower the yield of the target product but also impede the process of product recovery and purification. Therefore, elimination of byproduct formation to increase l-lactic acid yield is crucial. In our study, further disruption of the *adhB* and *ackA* genes based on strain RH08 resulted in a higher concentration, productivity, and yield of l-lactic acid, indicating that the carbon flux was channeled from ethanol and acetic acid production to l-lactic acid in strain RH15. The growth defect in the *pflA*-deleted strain RH12 has been observed in many other strains, such as *E. coli* [35], *Geobacillus thermoglucosidasius* [36], and *Klebsiella oxytoca* [37], and can be accounted for due to the high intracellular redox level rather than the reduced acetyl-CoA level, as PflA can catalyze the conversion of pyruvate to formic acid and acetyl-CoA simultaneously [38].

It has been emphasized that green processes using renewable biomass such as lignocellulosic hydrolysate are the trend in technological research and development; therefore, promoting these processes has become increasingly important. Thus far, the production of l-lactic acid has been investigated extensively in term of lignocellulosic biomass to decrease the use of edible biomass and to reduce the production cost [39, 40]. Table 4 lists the recent studies on l-lactic acid fermentation from mixed-sugars derived from lignocellulosic biomass. In batch fermentation, a relatively high l-lactic acid concentration (101.9 g/L) was acquired by *Pediococcus acidilactici* DQ2, though low lactic acid productivity (1.06 g/[L h]) was observed [41]. The highest productivity (3.28 g/[L h]) was observed in *B. coagulans* NBRC 12714, with an appreciable simultaneous concentration of l-lactic acid [10]. In fed-batch fermentation, the highest l-lactic acid titer (180 g/L) was achieved by *B. coagulans* strain P38, which also achieved an acceptable productivity of 2.40 g/[L h] [42]. There is no doubt that these studies have facilitated the commercialization of l-lactic acid production. However, the overall concentration and productivity of most systems for l-lactic acid production remain low, which cannot satisfy the requirements for large-scale industrial production. In the present study, our engineered strain RH15 was found to be an efficient producer for l-lactic acid production, and both the concentration and the productivity were competitive with most reported cases. Therefore, the efficient glucose and xylose utilization of the engineered *B. licheniformis* RH15 indicates its potential as a platform for producing other value chemicals or biofuels from lignocellulosic biomass.

**Table 4:** Overview of l-lactic acid production from lignocellulose-derived sugars

Microorganism	l-Lactic acid				Fermentation method	References
	Concentration (g/L)	Yield (g/g)	Productivity (g/[L h])	Optical purity (%)		
*Lactobacillus* sp. RKY2	42.0	0.95	6.70	ND	Continuous	[12]
*Bacillus* sp. XZL4	81.0	0.98	1.86	99.6	Batch	[13]
*B. coagulans* NL01	75.0	0.75	1.04	99.8	Fed-batch	[14]
*B. coagulans* MXL-9	40.2	0.58	0.54	99.5	Batch	[43]
*B. coagulans* IPE22	56.4	0.96	2.35	100	Repeated-batch	[5]
*B. coagulans* P38	180.0	0.98	2.40	100	Fed-batch	[42]
*Pediococcus acidilactici* DQ2	101.9	0.77	1.06	63.4	Batch	[41]
*B. coagulans* LA204	97.6	0.68	1.63	> 98	Fed-batch	[44]
*B. coagulans* 36D1	92.8	0.77	0.96	99.5	SSCF	[45]
*B. coagulans* P4-102B	91.8	0.78	0.82	99.5	SSCF	[45]
*B. coagulans* AD	35.2	0.95	3.69	ND	Continuous	[11]
*B. coagulans* NBRC 12714	98.3	0.95	3.28	> 99.5	Batch	[10]
*B. licheniformis* RH15	99.3	0.95	2.48	> 99.7	Fed-batch	This study

*SSCF* semi-continuous simultaneous saccharification and fermentation

## Conclusion

In this study, for the first time, *B. licheniformis* was engineered to produce l-lactic acid from lignocellulose-derived sugars. The glucose metabolic pathway was reconstructed to eliminate the CCR via abolishing the PTS system and activating the galactose transport route (GalP). The *xyl* operon was optimized to increase the xylose uptake rate by screening for the rate-limiting enzyme, xylose isomerase, in thermophilic bacteria. This “dual-channel” process enabled the engineered strain RH15 to produce l-lactic acid from glucose and xylose simultaneously. When the lignocellulosic hydrolysate was used as the substrate, 99.3 g/L l-lactic acid was produced, with a productivity of 2.48 g/[L h] and an optical purity of 99.7%. Thus, the engineered strain can serve as an efficient platform for chemical production from lignocellulosic biomass. This strategy might also be used to engineer other important strains to use inexpensive lignocellulose-derived sugars.

## Additional file

**Additional file 1: Figure S1.** The construction of gene knockout plasmids. **Figure S2.** The analysis of the stereoisomers of lactic acid produced by strain RH02. **Table S1.** Primers used in this study. **Text 1.** The codon-optimized sequences of *xylAs.*

## Abbreviations

CCR: carbon catabolite repression
GalP: galactose permease
PtsG: glucose transporter
GlcK: glucokinase
XylR: xylose repressor
PLA: polylactic acid
GRAS: generally regarded as safe
PTS: phosphotransferase system
GC: gas chromatograph
HPLC: high-performance liquid chromatography
AlsS: acetolactate synthase
AlsD: acetolactate decarboxylase
LDH: l-lactate dehydrogenase
XylA: xylulose isomerase
XylB: xylulose kinase
CRE: catabolite-responsive element
GN: Gram-negative
GP: Gram-positive
CSH: corn stover hydrolysate
IolT1: inositol permeases
XylT: xylose-proton symporter
PflA: pyruvate formate-lyase
AdhB: alcohol dehydrogenase
AckA: acetate kinase
